# Deep-Learning-Based Financial Message Sentiment Classification in Business Management

**DOI:** 10.1155/2022/3888675

**Published:** 2022-07-18

**Authors:** Chen Shao, Xiaochen Chen

**Affiliations:** ^1^School of Intelligent Engineering, Shandong Management University, Jinan 250357, China; ^2^School of Labor Relations, Shandong Management University, Jinan 250357, China

## Abstract

A deep-learning-based financial text sentiment classification method is proposed in this paper, which can provide a reference for business management. In the proposed method, domain adaptation is adopted to solve the common problem of insufficient labeled samples in the financial textual domain. Specifically, in the classification process, the seq2seq model is firstly adopted to extract the abstract from the financial message, which can reduce the influence of invalid information and speed up processing. In the process of sentiment classification, a bidirectional LSTM model is adopted for classification, which can more comprehensively make use of context information. Experiments are carried out to testify the proposed method through the open-source data set. It can be seen that the proposed method can effectively transfer from the reduced Amazon data set to the StockTwits financial text data set. Compared with the parameter-frozen-based method and the SDA-based method, the recognition rates have improved by 0.5% and 6.8%, respectively. If the target domain data set can be directly adopted for training, the recognition rate of the proposed method is higher than that of the SVM method and the LSTM method by 8.3% and 4.5%, respectively.

## 1. Introduction

Text-based sentiment classification has significant importance for business management. The effect of sentiment classification is mainly twofold. Firstly, through sentiment analysis of current financial texts, the current economic situation can be revealed, so as to adjust corresponding corporate strategies. Secondly, the comments on the corporate's products and the corporate itself can be performed for sentiment classification, so as to provide references for the corporate's products or the corporate itself.

Among the mentioned two aspects, sentiment analysis based on financial texts has a particularly significant effect on business management. For example, by extracting important features from financial texts, including financial news, financial comments, and financial-theme-related social networks, it is possible to perceive the emotions of the crowd and predict the financial or economic situation trends. This can also provide references for the strategic team, including making the financing strategy, management strategy of the corporate, and so on. In this way, as information is obtained from a large amount of text data from a large crowd, the influence of subjective factors from the management personnel can be effectively eliminated. Therefore, sentiment analysis from financial texts has become a research hotspot in recent years.

Currently, there already exists extensive research for sentiment analysis of texts. There are mainly two types of methods. The first type is the traditional machine learning based methods, and the other is the deep-learning-based methods. However, no matter what type of method it is, effective mathematical representations of texts are needed at first. For early text representation methods, the texts are regarded as merely a set of words with the same weight, such as the bag-of-words (BoW) method [1–3], which has ignored the underlying grammar and sequences of words. Similar methods include the term frequency–inverse document frequency (TF-IDF) method [4–6], which goes a step further and takes into account the different importance of different words. In this method, it is believed that the importance of words is proportional to the frequency of occurrence in the text and inversely proportional to the frequency of occurrence in the corpus. Currently, the most widely adopted method for text representation is the word2vec method [7–9]; the main idea is to use vectors to represent different words. For both the representational vector space and the real word meaning space, the measures of distance between words are similar. In the word2vec method, the research focus is on how to find a mapping from words to vectors so that the similarity of words in the vector space is preserved. The methods for establishing this mapping relationship include the continuous bag-of-words (CBOW) model [10, 11] and the skip-gram model [12, 13], which are both trained through the corpus to obtain the representational vectors of different words. In this context, this process is also referred to as a pretraining process, and currently, there already exists vector representations pretrained adopting a rich corpus.

For the first type of sentiment classification method mentioned above, the sentiment of texts is analyzed by adopting traditional classifiers, such as support vector machines (SVM), random forests, multinomial naïve Bayes (mNB), and other models. The related literature on these methods are [14–16]. In these traditional methods, the types of classifiers are different, while the features adopted are similar, which are not fully utilized, resulting in a limited recognition rate. For the second type of method, as deep-learning-based techniques can extract more abstract or high-level features from the text, often a better classification performance can be reached.

In this paper, by estimating the current economic situation through financial texts, business management can be improved. However, for such a purpose, the use of deep learning for sentiment classification from financial texts has two main problems: (1) the problem of insufficient amount of labeled financial texts and (2) the problem of establishing an efficient and effective model to improve the classification accuracy. Existing methods are then introduced following the logic of how to solve the mentioned two main problems.

In terms of sentiment analysis from financial texts, currently there exists an obvious problem, which is the lack of sufficient labeled financial texts. For this problem, a relatively straightforward solution is to adopt the labeled samples from other textual domains to make up for the lack of labeled financial textual samples. Then transfer learning can be applied for that. In literature [17], fine tuning is proposed for transfer learning from other textual domains to the financial textual domain. In this method, after a model is trained with a large number of labeled samples, the parameters of some layers are then frozen, mostly the shallow feature extraction layers in the front, and then other parameters are fine-tuned adopting a small number of labeled samples in the financial text domain. Noting that in this method, only the parameters of the abstract classification layer are fine-tuned to achieve transfer learning purposes. In this method, since the feature extraction parameters of the shallow layers are frozen, and new features cannot be obtained for the classification of new data domains, the transfer learning performance is often limited. In [18], a combination of supervised and unsupervised methods is proposed. Specifically, the input samples are dimensionally reduced adopting the stacked denoising autoencoder (SDA) to obtain the shared feature vector among different input domains, and then the sentiment is estimated by another classifier. In this method, as the labeled samples are not adopted in the feature extraction process, the capability of this method is limited in terms of feature extraction. In general, although this method has comparatively good generality among different sample domains, its classification performance is limited. The authors in [19] have proposed an adversarial learning method to solve the problem of an insufficient number of labeled samples. In this adversarial network, there is a compromise between the loss of sentiment classification and the loss of domain classification. In [20], the idea of active learning is adopted, and the number of labeled samples required in the target domain in training are directly reduced by the method of active learning. However, in this active learning method, the reduction of labeled samples is only validated terms without active learning, and a large number of labeled samples are still needed.

In addition to solving the problem of insufficient labeled samples, it is also necessary to select a suitable model for textual sentiment classification. In [21], it is proposed that in order to better perform sentiment classification, multiple sources of information can be used, such as text information, images, or even videos. This is also referred to as multimodal classification. The method of multimodal classification can be considered as a type of methods for solving the problem of lack of training samples. The idea is to add more types of information other than textual information. However, to make it work, there still needs more training information. In literature [22, 23], the textual features and visual features are fused through the attention-based recurrent neural network (RNN) model and the adversarial network model, respectively, which can improve the classification accuracy compared to the single information source. In [24], it is proposed to further apply multimodal classification to the field of fake information detection. The two different feature vectors are merged through the multimodal compact bilinear pooling (MCBP) method, which can effectively fuse the two kinds of information for classification. In this paper, since most of the samples for financial sentiment analysis only contain textual information, only the unimodal sentiment classification (from textual information) is studied. Existing classification models can also be divided into two categories, convolutional neural network (CNN) based models and RNN-based models. The related literature include [25–29]. Generally speaking, among the two types, the RNN-based models generally have better classification performance due to better utilization of contextual information.

A deep-learning-based financial text sentiment classification method is proposed in this paper, which can provide a reference for business management. In the proposed method, domain adaptation is adopted to solve the common problem of insufficient labeled samples in the financial textual domain. A subnetwork for distinguishing domains is added to the common sentiment classification network, and domain-related loss is also added to the overall cost function. In the proposed method, sentiment classification of financial text is possible without labeled financial text samples (i.e., target domain sample labels). In addition, in the classification process, the seq2seq model is firstly adopted to extract the abstract from the financial message, which can reduce the influence of invalid information and speed up the processing. In the process of sentiment classification, a bidirectional (long short-term memory) LSTM model is adopted for classification, which can more comprehensively make use of context information. In addition, an attention mechanism is also added to ensure that the information usage is comprehensive, while critical information are more weighted. Experiments are carried out to testify the proposed method through the open-source data set. It can be seen that the proposed method can effectively transfer from the reduced Amazon data set to the StockTwits financial text data set. Compared with the parameter freezing method and the SDA-based method, the recognition rates have improved by 0.5% and 6.8%, respectively. If the target domain data set can be directly adopted for training, the recognition rate of the proposed method is higher than that of the SVM method and the LSTM method by 8.3% and 4.5%, respectively.

## 2. Methods

The flow chart of the proposed method in this paper is shown in Figure 1. It can be seen that the proposed method can be divided into three parts. The first part is to adopt the seq2seq model to extract the abstract of the message. Here, the extracted abstract is of fixed length. Moreover, the seq2seq model adopted in this paper is not trained in the implementation of the method but is already pretrained by adopting existing rich corpus. In our method, it is directly put to use as a general abstract extraction model. Therefore, the impacts of different textual domains on abstract extraction have not been taken into consideration here. After the abstract extraction, a highly summative abstract of the text is obtained, which can reduce the influence of invalid information on classification. The second part of the proposed method contains a feature extraction subnetwork based on the bidirectional LSTM model, which can use the extracted abstract information (also the output of the seq2seq model) to further summarize the abstract. The output is a feature vector, which can be used for both sentiment classification and the domain classification. There are two domains here: the source domain and the target domain. The source domain refers to a large number of texts (mainly product comments in our implementation) with sentiment classification labels, and the target domain refers to financial texts, which is not labeled. The third part contains two paralleled classification subnetworks, the sentiment classification subnetwork and the domain classification subnetwork. The sentiment classification subnetwork is adopted for the final text sentiment classification, and the sentiment classification cost is constructed from the labeled textual samples. The domain classification subnetwork is adopted to distinguish sample domains, with the domain discrimination cost function. The proposed method in this paper is introduced as follows according to the three parts mentioned above. Noting that here the domain adaptation can be considered as a framework of the proposed framework. With different losses, including the sentiment classification loss and the domain classification loss added to the proposed method, domain adaptation is realized. However, for the seq2seq-model-based abstraction part, it is a standalone processing flowing. In our implementation, the extracted abstract is of fixed length. Moreover, the seq2seq model adopted in this paper is not trained in the implementation of the method but is already pretrained by adopting existing rich corpus.

### 2.1. Abstract Extraction Based on the Seq2seq Model

The seq2seq model adopted in this paper is described in Figure 2. The seq2seq model is often adopted in the field of automatic translation in natural language processing (NLP), where the input is of one language and the output is another language. In our paper, the pretrained seq2seq abstract extraction model is directly adopted; the input is the descriptive text; and the output is a fixed-length abstract. Since the application of the seq2seq model in abstract extraction has already been widely studied, only some key points are described herein.

As shown in Figure 2, the basic structure of the seq2seq model is encoder-decoder-based. The context vector is the connection between the encoder and the decoder, which is the output of the encoder and the input of the decoder. This vector can be regarded as an effective summary of the input according to the encoder, which contains the contextual information of the input sequence. Generally speaking, both the encoder and decoder contain long short-term memory (LSTM), so as to keep the memory of the sequence. However, the pure encoder-decoder structure can suffer from the loss of sequence information. When the input sequence is long and the dimension of the context vector is low, more information can be neglected from the encoder. This can lead the decoder to work abnormal due to the loss of key information.

To solve the problem, a straightforward idea is to add different importance to the input sequence. Therefore, attention-based encoder-decoder model is proposed in [30]. In the attention-based model, the context variable is the weighted average of the encoder output hidden variables *h*_*j*_ and weights *w*_*ij*_, which can be expressed as follows:

(1) $$\begin{array}{c} cv_{i}=\sum_{j=1}^{T}w_{ij}h_{j}. \end{array}$$

The weights of different hidden variables *w*_*ij*_ are calculated according to *e*_*ij*_. *e*_*ij*_ is jointly determined by the hidden variables of the encoder and the decoder at different times (where *h*_*j*_ denote the output hidden variables of the encoder and *c*_*j*_ denote the output hidden variables of the decoder) according to the score function get_score(.). The score function is also called the alignment function, and the dot product of the two hidden vectors is directly applied in this paper.

(2) $$\begin{array}{c} w_{ij}=\frac{\text{exp}e_{ij}}{\sum_{k=1}^{T}\text{exp}e_{ik}},\\ e_{ij}=\text{get\_score}\left(c_{j},h_{j}\right),\\ \text{get}\_\text{score}\left(.\right)\equiv \left(.\right) \end{array}$$

In the seq2seq model, the output is a series of sequences and their respective probabilities. Usually, in order to avoid the probability of accidental output, only one sequence is finally taken as the maximum probability output, and the BeamSearch algorithm can be used to obtain the sequence output with the maximum overall probability.

### 2.2. Feature Extraction Subnetwork Based on Bidirectional LSTM

The proposed feature extraction subnetwork based on bidirectional LSTM is applied to extract the information in the abstract and to generate the corresponding feature vector, which can be adopted for the subsequent sentiment classification and the domain classification. Note that here the feature extraction subnetwork is different from a common feature extraction network. It not only needs to take into account the extraction of sentiment classification-related features but also the features that can distinguish source or target domain data samples. Its basic structure is shown in Figure 3.

According to the descriptions in the paper [31], the model of bidirectional LSTM can extract more comprehensive features because the extracted feature is related to the total semantic information. By adding an attention mechanism on this basis, it can be ensured that the key information is retained in a focused manner as well as the comprehensiveness of the information. In Figure 3, *F* represents the final state of the bidirectional LSTM model, that is, the addition result of the state values of the forward and backward hidden layers.

The calculation process of the attention probability distribution and the calculation process of the final feature vector with the attention mechanism are as follows, which generally include two main steps:

(3) $$\begin{array}{c} a_{n}=\frac{\text{exp}\left(h_{n}^{\prime }\right)}{\sum_{i=1}^{N}\text{exp}\left(h_{i}^{\prime }\right)},\\ h_{n}^{\prime }=h_{n}^{T}UF, \end{array}$$

where *a*_*n*_ denotes the attention probability distribution of the hidden layer unit at time *n*, *h*_*i*_′ denotes the input sequence, and *U* denotes the weighting matrix. *h*_*n*_ denotes the sum of the bidirectional hidden layer state values at the time *n*. With the bidirectional LSTM model, the feature vector *F* can be obtained. The difference between the abstract extraction model and the feature extraction model is as follows. For the abstract extraction process, the model is just based on a one direction seq2seq model with an encoder-decoder structure. However, for the feature extraction process, the model is bidirectional LSTM-based. The model of bidirectional LSTM can extract more comprehensive features because the extracted feature is related to the total semantic information.

### 2.3. Sentiment Classification Subnetwork and Domain Classification Subnetwork

After the feature vector is obtained, it can be adopted for sentiment classification and domain classification by the sentiment classification subnetwork and the domain classification subnetwork, respectively. In this paper, the sentiments in the financial text domain are bullish and bearish, respectively, and the different domains are the financial text domain and other data domains, respectively.

In this paper, the structures of the sentiment classification subnetwork and the domain classification subnetwork are shown in Figures 4 and 5, respectively. It can be seen that the two subnetworks have similar structures. The only difference is that the domain classification subnetwork has an additional layer of reverse gradient layer in the beginning, which will be introduced later. The mutual structure in both the sentiment classification subnetwork and the domain subnetwork is introduced as follows, including a fully connected layer and a softmax layer. The operation of the softmax layer is as follows:

(4) $$\begin{array}{c} l_{i}=\frac{o^{i}}{\sum_{j=1}^{N}o^{j}}, \end{array}$$

where *o*^*i*^ represents the component of the *i*th dimension in the input vector, *l*_*i*_ denotes the output probability of the *i*th dimensional component, and *N* represents the total number of classes.

The purpose of the domain classification subnetwork is to distinguish whether the data samples originated from the financial textual domain. The addition of the reverse gradient layer mentioned above can achieve the following effects: (1) enabling the domain classification subnetwork to distinguish whether it originated from the financial textual domain, (2) while making the features in the feature extraction subnetwork unable to extract features that are sensitive to specific domains. The mentioned effects can achieve the purpose of transfer learning. The inverse gradient layer can be expressed as follows:

(5) $$\begin{array}{c} F\left(s\right)=s,\\ \frac{\partial F\left(s\right)}{\partial s}=-\eta I, \end{array}$$

where the function **F**(.) denotes the function of forward propagation and **s** denotes the input vector. In the forward propagation process of the reverse gradient layer, the layer has no special operation on the input data sample. However, during training, the gradient of back propagation is reversed and linearly reduced in this layer. The addition of the reverse gradient layer has enabled domain classification subnetwork training while making the feature extraction subnetwork unable to extract features related to domain classification. Therefore, the purpose of transfer learning can be achieved.

The proposed network has two cost functions in the training process, namely the sentiment classification cost function and the domain classification cost function. The two cost functions have similar structures, and they are both cost functions based on cross-entropy, which are

(6) $$\begin{array}{c} {\text{Loss}}_{1,i}\left(.\right)=-\sum d_{1,i}\text{log}l_{1,i},\\ {\text{Loss}}_{2,j}\left(.\right)=-\sum d_{2,j}\text{log}l_{2,j}, \end{array}$$

where the subscript 1 is sentiment classification related and 2 is domain classification related; Loss(.) denotes the cost function; *l* denotes the corresponding output through the softmax layer, that is, the probability of the corresponding label; and *d* denotes the real label (i.e., the real label vector representation after one-hot encoding). The subscripts *i* and *j* represent the index of the training samples.

Then the final cost function can be expressed as the sum of two subcost functions as follows:

(7) $$\begin{array}{c} {\text{Loss}}_{\text{all}}\left(.\right)={\text{Loss}}_{1}\left(.\right)-\eta {\text{Loss}}_{2}\left(.\right) \end{array}$$

A minus sign and a linear parameter *η* are added to the domain classification cost function, which is equivalent to the operation of the reverse gradient layer mentioned above. Setting the cost function in this way is equivalent to only adding the reverse operation of the gradient during the training process, without affecting the forward inference process.

## 3. Results and Discussion

As transfer learning is needed in this paper, so data sets of source and target domains are both required. To validate the proposed method in this paper, the selected data sets the source and target domains are both open-sourced. The selected source domain is the classic reduced Amazon data set. The data set comprises comments of four products: books, DVDs, electronics, and kitchen appliances. Each category contains 2,000 labeled reviews, including 1,000 positive reviews and 1,000 negative reviews, each accounting for 50%. We chose the financial social network StockTwits as the target domain data set. The labels of this data set are bullish and bearish. In order to facilitate domain adaptation, we correspond bullish to positive labels in the reduced Amazon data set and bearish to negative labels. Although we have not used the labels of the target domain during training, the labels of the target domain are actually known and can be adopted for statistical purposes. For the above data sets, the training set and the test set are split according to 70% and 30%.

Since the proposed method can be divided into two aspects, the first is based on transfer learning between different data domains; the second is abstract extraction by seq2seq; and then the recognition is based on bidirectional LSTM. Therefore, here the experimental comparison is also set up according to these two aspects.

### 3.1. Comparison of Transfer Learning Methods

For comparisons of transfer learning methods, the SDA-based method and the parameter-frozen-based method described above are selected for comparison. Note that among these methods, the proposed method in this paper and the SDA-based method can both be regarded as an unsupervised transfer learning method, which does not require any labeled samples from the target domain during training. The method of parameter frozen is semisupervised, which requires a small number of labeled samples from the target domain.

The comparison results of the three methods are shown in Figure 6 and Table 1. It can be seen that the accuracy of domain classification of the proposed method has reached 61.2%. Compared with the parameter-frozen-based method and the SDA-based method, the recognition rate has improved by 0.5% and 6.8%, respectively. The results have fully illustrated the effectiveness of the proposed method in textual domain classification, which can provide an effective solution for the problem of the small number of labeled samples in the target domain mentioned above. Although the improvement is not obvious compared with the parameter frozen method, it should be noted that the parameter frozen method has adopted a small number of labeled samples in the target domain, while the proposed method has not. Noting that the results here are already the overall results. The comparisons in the next part are made without considering the domain adaptation framework so that the effects of other factors including the abstract extraction and the bidirectional LSTM model can be tested.

### 3.2. Comparison of Classification Methods

After the transfer learning part is verified, the recognition effect of the proposed seq2seq abstract extraction + bidirectional LSTM feature extraction framework will be tested. In order to be able to compare with other recognition methods, in this section, we have skipped the source domain and have directly taken the labeled samples in the target domain for training. Here, the proposed method in this paper is also compared with the two recognition methods mentioned above. The first method is a traditional SVM-based method without deep learning. The second method is based on LSTM, which does not include the abstract extraction part and directly adopts the original message as the input. The comparison results are shown in Figure 7 and Table 2. It can be seen that the recognition rate of the proposed method in this paper has reached 80.7%. Compared with the SVM method and LSTM method, it has improved by 8.3% and 4.5%, respectively.

In order to further study the characteristics of the proposed method, the contribution of the abstract extraction and bidirectional LSTM factors to the final recognition accuracy is also looked into. There are three cases for comparison: (1) adding abstract extraction and bidirectional LSTM feature extraction (the proposed), (2) without abstract extraction, only with bidirectional LSTM feature extraction, (3) with abstract extraction and with ordinary LSTM-based feature extraction, and (4) without abstract extraction and with ordinary LSTM-based feature extraction.  Table 3 has listed the different recognition rates in the four cases. It can be seen that the factors of abstract extraction and bidirectional LSTM both have a significant impact on improving recognition accuracy. Compared with cases 2, 3, and 4, the recognition accuracy of case 1 has improved by 3.6%, 3.2%, and 4.5%, respectively.

## 4. Conclusions

A deep-learning-based financial text sentiment classification method is proposed in this paper, which can provide a reference for business management. The proposed method has adopted the domain adaptation framework to solve the common problem of insufficient labeled samples in financial text classification. Specifically, in the classification process, the seq2seq model is first adopted to extract the abstract from the financial message. Then, a bidirectional LSTM model is adopted for classification, which can more comprehensively make use of context information. Experiments are carried out to testify the proposed method through the open-source data set. It can be seen that the proposed method can effectively transfer from the reduced Amazon data set to the StockTwits financial text data set. Compared with the parameter-frozen-based method and the SDA-based method, the recognition rates have improved by 0.5% and 6.8%, respectively. If the target domain data set can be directly adopted for training, the recognition rate of the proposed method is higher than that of the SVM method and the LSTM method by 8.3% and 4.5%, respectively. In addition, results have also shown that the factors of adding abstract extraction and adopting the bidirectional LSTM model can both be effective in improving performance.

## Figures and Tables

**Figure 1:** The processing flowchart of the proposed method in three parts.

**Figure 2:** The encoder-decoder structure of the adopted seq2seq model.

**Figure 3:** The feature extraction subnetwork based on the bidirectional LSTM model.

**Figure 4:** The structure of the sentiment classification subnetwork.

**Figure 5:** The structure of the domain classification subnetwork.

**Figure 6:** The histogram of the average recognition rate of different methods.

**Figure 7:** Comparison of the classification accuracy of the proposed method, the traditional SVM method, and the LSTM-based method.

**Table 1:** Comparison of average recognition rates of different methods.

Method	Accuracy (%)	Improvement (%)
Proposed method	61.2	—
SDA-based method	57.3	6.8
Parameter-frozen-based method	60.9	0.5

**Table 2:** Comparison of the classification accuracy of the proposed method, the traditional SVM method, and the LSTM-based method.

Method	Accuracy (%)	Improvement (%)
Proposed method	80.7	—
SVM-based method	74.5	8.3
LSTM-based method	77.2	4.5

**Table 3:** The comparisons of the proposed method and the other three cases.

Situation	Accuracy (%)	Improvement (%)
Case 1	80.7	—
Case 2	77.9	3.6
Case 3	78.2	3.2
Case 4	77.2	4.5

## Data Availability

The data adopted in the paper are available at https://stocktwits.com.
